RETRACTED

# Meta-Analysis of the Effect of Glucocorticoids on Adult Acute Respiratory Distress Syndrome

**DOI:** 10.1155/2022/4020489

**Published:** 2022-08-10

**Authors:** Haopeng Wu, Li Chen, Hui Lin, Fen Sheng

**Affiliations:** ^1^Department of Emergency, Taizhou First People's Hospital, Taizhou 318020, Zhejiang, China; ^2^Department of Respiratory and Critical Care Medicine, Enze Hospital, Taizhou Enze Medical Center (Group), Taizhou 318050, Zhejiang, China; ^3^Department of General Practice, Taizhou First People's Hospital, Taizhou 318020, Zhejiang, China; ^4^Department of Respiratory and Critical Care Medicine, Taizhou First People's Hospital, Taizhou 318020, Zhejiang, China

## Abstract

**Objectives:**

The aim of this study is to investigate the effect of glucocorticoids in adult patients with acute respiratory distress syndrome (ARDS) by meta-analysis.

**Methods:**

PubMed, Cochrane Library, Embase, CNKI, Wanfang Database, and Chinese Biomedical literature database were searched. A randomized controlled trial (RCTS) on glucocorticoid therapy in adult patients with ARDS was conducted from the time of database construction to December 2021. The content is about the randomized controlled trial (RCT) of glucocorticoid treatment for adult patients with ARDS, without limiting the dose and course of glucocorticoid treatment. The quality of the included RCTS was evaluated by using the bias risk assessment tool of the Cochrane Collaboration network, and the basic information, clinical features, and target outcomes of the literature were extracted. The effects of glucocorticoids on mortality and oxygenation index (PaO_2_/FiO_2_) in adult ARDS patients were evaluated by meta-analysis.

**Results:**

A total of 1,441 ARDS patients in 10 RCTs were finally included, including 734 patients in the glucocorticoid treatment group (hormone group) and 707 patients in the conventional treatment group (control group). The 10 studies included have a good overall design and high quality. Compared with controls, glucocorticoid use was significantly associated with a decrease in mortality in adult ARDS patients (relative risk (RR) = 0.73, 95% confidence interval (95% CI) = 0.59–0.90, *P* = 0.003). Analysis showed that glucocorticoids significantly reduced the mortality in ARDS patients treated with medium and low doses of steroids (RR = 0.73, 95% CI = 0.58–0.92, *P* = 0.007). In patients with early administration of steroids, intervention with glucocorticoids was significantly associated with the decreased mortality in adult ARDS patients compared with controls (RR = 0.74, 95% CI 0.56–0.99, *P* = 0.04). Among patients with more than 7 days of hormone therapy, treatment with glucocorticoids was significantly associated with decreased mortality in adult ARDS patients (RR = 0.66, 95% CI = 0.50–0.88, *P* = 0.005) compared with controls. Glucocorticoids tended to improve PaO_2_/FiO_2_ in adult ARDS patients compared with controls, but the difference was not statistically significant (weighted mean difference (WMD) = 11.60, 95% = CI = 15.02–38.22, *P* = 0.39).

RETRACTED

**Conclusion:**

Glucocorticoid therapy can reduce mortality in adult ARDS patients, and the benefit is more pronounced in patients with medium- and low-dose hormone therapy, early hormone administration, and hormone therapy for more than 7 days. However, no improvement in PaO_2_/FiO_2_ by glucocorticoid treatment was found, which needs to be confirmed by further studies.

## 1. Introduction

Acute respiratory distress syndrome (ARDS) is an inflammatory lung injury disease caused by various causes and characterized by increased permeability of pulmonary capillary endothelial cells and alveolar epithelial cells [1], which is mainly characterized by respiratory distress and severe hypoxemia. Lung involvement is common in severe pneumonia or systemic inflammatory reaction [2]. ARDS is a serious organ dysfunction disease with an estimated mortality of up to 40% in hospital. Timely diagnosis and treatment can effectively reduce the mortality of patients [3]. Studies have shown that excessive inflammatory response may be an important cause of high mortality [4]. Inflammatory factors, including interleukin-1, interleukin-6 and C-reactive protein, mediate lung epithelial barrier damage and increased vascular permeability and promote the development of ARDS [5]. The effective treatment methods for ARDS are mainly protective lung ventilation strategy and prone position ventilation [6], but there is still a lack of effective drug treatment. Glucocorticoids are potent anti-inflammatory drugs commonly used in clinical practice and have the effects of antifibrosis and improving physical stress capacity [7]. Glucocorticoids may improve the prognosis of ARDS patients by reducing the levels of inflammatory factors and inhibiting the activation of inflammatory processes [8]. Recent studies suggest that small doses of hormone (methylprednisolone ≤2 mg·kg^−1^·D^−1^) can effectively reduce the level of inflammatory factors in ARDS patients, improve lung function, reduce the use of ventilators, and reduce the mortality of ARDS patients [9]. However, it has also been shown that glucocorticoids do not reduce the risk of death in ARDS patients [10]. Therefore, there are still controversies about the results of clinical studies in the use of glucocorticoids in the treatment of ARDS, and the timing, dose, and course of hormone use remain elusive. The aim of this study was to evaluate the effect of glucocorticoids on the mortality and oxygenation index (PaO_2_/FiO_2_) in adult ARDS patients through a meta-analysis of published randomized controlled trials (RCTs) and to investigate the appropriate timing, dose, and course of hormone application.

RETRACTED

## 2. Data and Methods

### 2.1. Literature Retrieval

A literature search was conducted in PubMed, Cochrane Library, Embase, CNKI, Wanfang Database, and Chinese Biomedical literature database, and RCT studies on the treatment of adult ARDS patients with glucocorticoids published from the establishment of the database to December 2021 were included. English search terms include “acute respiratory distress syndrome,” “acute lung injury,” “ARDS,” “ALI,” “glucocorticoids,” “corticosteroid,” “methylprednisolone,” “hydrocortisone,” “dexamethasone,” and “hexadecadrol”; read the list of reviews and references searched for articles that meet the criteria.

### 2.2. Inclusion Criteria and Exclusion Criteria

Inclusion criteria were as follows: (1) the study design was an RCT; (2) patients aged ≥18 years, regardless of race and gender; (3) a definite diagnosis of ARDS, regardless of specific etiology; (4) the study included a control group receiving placebo or standard treatment with glucocorticoid intervention, and the study provided data on the starting time, dose, course of treatment, mortality in the two groups, and PaO_2_/FiO_2_ of hormone therapy. The exclusion criteria were as follows: (1) animal studies, or studies in infants and children; (2) glucocorticoids for prevention rather than treatment of ARDS; (3) no diagnostic criteria for ARDS were given in the studies; (4) no required data were provided in the studies; and (5) types of literature such as conference abstracts, reviews, and case reports.

### 2.3. Data Extraction and Quality Assessment

Two independent investigators extracted data on the following variables from the included studies: author, year of publication, study design, sample size of both groups, demographic data, initiation of glucocorticoid therapy, hormone dose, hormone course, mortality, and PaO_2_/FiO_2_, etc. The quality of the included RCTS was evaluated using the Cochrane Collaboration network bias risk assessment tool. A third evaluator worked together to resolve differences.

### 2.4. Outcome Indicators

Main outcome measure is mortality; secondary outcome measure is oxygenation index (PaO_2_/FiO_2_). Subgroup analysis was performed according to glucocorticoid initiation time, dose, and duration. Early administration of hormones was defined as the first 7 days of ARDS diagnosis and late administration as 7 days after ARDS diagnosis. Medium- and low-dose glucocorticoids were defined as methylprednisolone ≤2 mg·kg^−1^·d^−1^, and high-dose was defined as methylprednisolone >2 mg·kg^−1^·d^x1^, which was converted to an equivalent dose of methylprednisolone based on 20 mg hydrocortisone and 0.75 mg dexamethasone equivalent to 4.0 mg methylprednisolone.

RETRACTED

### 2.5. Statistical Analysis

Mean ± standard deviation was used to represent continuous variables. Relative risk (RR) and 95% confidence interval (CI) were used to analyze mortality. Weighted mean difference (WMD) and 95% CI were used to analyze PaO_2_/FiO_2_. *χ*^2^ test was used to determine the heterogeneity between studies. When *P* ≥ 0.1 and *I*^2^ ≤ 50%, the heterogeneity between studies was considered small, and the fixed-effect model was used. When *P* < 0.1 and *I*^2^ > 50%, the random effect model was used. Bilateral *P* < 0.05 indicated a statistically significant difference, and RevMan 5.3 software was used for meta-analysis.

## 3. Results

### 3.1. Literature Screening

As shown in Figure 1, the total number of screened articles was determined to be 5482 after database search, 2587 duplicate articles were excluded, and 2335 articles were excluded by reading the article title and abstract. Five hundred and sixty articles were reviewed in full text, and a total of 550 articles without outcome measures or only conference abstracts were excluded. Finally, a total of 10 RCTs were included in the analysis [11–20].

### 3.2. Clinical Features Included in the Study

As shown in Table 1, a total of 1,441 ARDS patients were included, including 734 in the steroid group and 707 in the control group. Patients in both groups received standard treatment such as mechanical ventilation, expectorant, anti-asthmatic, and anti-infective. The mean age ranged from 47.0 to 66.6 years in the hormone group and from 49.0 to 64.3 years in the control group. The types of hormones used included hydrocortisone, methylprednisolone, and dexamethasone. The doses of hydrocortisone used were 50 mg/6h and 240 mg/day. Methylprednisolone was used at doses of 1 mg/kg/day, 2 mg/kg/day, 120 mg/day and 1 g/day. Dexamethasone was used at doses of 1 mg/kg/day and 20 mg/day. The duration of hormonal therapy ranged from 1 day to 32 days.

### 3.3. Quality Evaluation of Included Studies

As shown in Figure 2, the overall design of the study was scientific and of high quality. Four RCTs were low-risk. Four RCTs had unclear results of selective reports and bias from other sources. One RCT had unclear grouping hidden, unclear selective report results, and unclear bias from other sources. The remaining 1 RCT had an unclear random grouping method, unclear grouping hiding, unclear selective report results, and unclear bias from other sources.

RETRACTED

### 3.4. Effects of Glucocorticoids on Mortality in Adult ARDS Patients

Figure 3 includes a total of 10 studies showing the effect of glucocorticoids on mortality in adults with ARDS. Compared with the control group, glucocorticoid use was significantly associated with reduced mortality in adult ARDS patients (RR = 0.73, 95% CI = 0.59–0.90, *I*^2^ = 44%, *P*=0.003).

### 3.5. Subgroup Analysis of Effects of Glucocorticoids on Mortality in Adult ARDS Patients

As shown in Table 2, the analysis was performed according to the hormone dose, the starting time of the hormone, and the duration of the hormone. Among patients treated with medium-dose and low-dose steroids, glucocorticoids could significantly reduce the mortality of ARDS patients (RR = 0.73, 95% CI = 0.58–0.92, *I*^2^ = 34%, *P* = 0.007). Among patients treated with high-dose steroids, glucocorticoids tended to reduce mortality, but the difference was not statistically significant (RR = 0.70, 95% CI = 0.36–1.38, *I*^2^ = 82%, *P* = 0.31). In patients with early hormone administration, glucocorticoid intervention was significantly associated with the decreased mortality in adult ARDS patients compared with controls (RR = 0.74, 95% CI = 0.56–0.99, *I*^2^ = 55%, *P* = 0.04), and a trend toward decreased mortality could also be observed in patients with late hormone administration (RR = 0.68, 95% CI = 0.47–0.99, *I*^2^ = 38%, *P* = 0.05). In patients treated with corticosteroids for more than 7 days, it can be seen that compared with the control group, there was a significant correlation between the treatment of glucocorticoids and the mortality of adult ARDS patients, but this correlation was not observed in patients treated with corticosteroids for less than 7 days.

### 3.6. Effects of Glucocorticoids on PaO_2_/FiO_2_ in Adult ARDS Patients

Figure 4 includes a total of 8 studies showing the effect of glucocorticoids on PaO_2_/FiO_2_ in adult ARDS patients. Compared with the control group, glucocorticoids tended to improve PaO_2_/FiO_2_ in adult ARDS patients, but the difference was not statistically significant (WMD = 11.60, 95% CI, 15.02 to 38.22, *I*^2^ = 97%, *P*=0.39).

## 4. Discussion

In this study, glucocorticoid use was significantly associated with the reduced mortality in adults with ARDS compared with the control group. Notably, benefits were more pronounced in patients who received low doses of hormone therapy, early hormone administration, and hormone therapy for longer than 7 days. In addition, compared with the control group, glucocorticoids tended to improve PaO_2_/FiO_2_ in adult ARDS patients, but the difference was not statistically significant.

RETRACTED

The pathophysiological changes of ARDS are some pathogenic factors causing increased vascular permeability and exudation of large amounts of fluid into the alveolar space causing pulmonary edema, while alveolar epithelium is damaged, resulting in a reduced pulmonary surfactant synthesis and increased pulmonary surface tension, both of which act together to cause hypoxemia [1]. The activation of inflammatory processes and the involvement of inflammatory factors further promote the development of ARDS [21]. At present, the mortality rate of ARDS is still high, and timely and effective treatment measures can improve the prognosis of patients [22].

A meta-analysis involving five studies showed that glucocorticoid treatment may be associated with a decreasing trend in mortality, but the sample size of the study was small [23]. This study included 1,441 patients with ARDS, and pooled analysis showed that glucocorticoid use was significantly associated with a decrease in mortality in adult ARDS patients (RR = 0.73, 95% CI = 0.59–0.90, *P*=0.003). However, other studies have shown that short-term and high-dose glucocorticoid therapy may even worsen the risk of ARDS or patients with ARDS [24]. The inconsistencies in the abovementioned studies may be attributed to patient population characteristics, sample size, and hormone dose and duration.

Glucocorticoids have a potent effect and can indirectly play a role by inhibiting the activation of inflammatory processes, including inhibiting the gene transcription of proinflammatory factors, inhibiting the expression of inducible nitric oxide, and promoting the production of interleukin-10 and interleukin-4 [25]. In addition, glucocorticoids can also improve coagulation and inhibition response, thereby normalizing the ventilation/blood flow ratio [26]. Based on the abovementioned effects of hormones, they should theoretically significantly improve the oxygenation index in ARDS patients, but the clinical results are inconsistent. This study found that glucocorticoids tended to improve PaO_2_/FiO_2_ in adult ARDS patients compared with the control group, but the difference was not statistically significant (WMD = 11.60, 95% CI, 15.02 to 38.22, *P*=0.39). This suggests that glucocorticoids may have other possible ways to reduce the mortality.

Initiation time, dose, and course of glucocorticoid therapy are also important factors affecting the prognosis of adult ARDS patients [27]. Similar to the results of this study, some studies suggest that early administration and low dose administration of glucocorticoids can significantly improve the prognosis of ARDS patients [10]. In addition, glucocorticoid treatment was significantly associated with reduced mortality in adult ARDS patients treated for more than 7 days compared with the control group (RR 0.66, 95% CI 0.50–0.88, *P*=0.005). However, no such correlation was observed in patients who received hormone therapy within 7 days (*P* > 0.05).

RETRACTED

This study also has the following limitations: (1) The analysis of the literature can only provide exploratory results but does not suggest a clear correlation, and further inflammation is needed in the future. (2) The safety of glucocorticoids was not evaluated in this study, and previous studies suggest that glucocorticoids may increase the risk of hyperglycemia and new infection [28]. (3) Meta-analysis can only suggest a correlation relationship, and a large sample of RCTs is needed in the future to further evaluate the role of glucocorticoids in adult ARDS patients.

In summary, glucocorticoid therapy reduces the mortality in adult ARDS patients, and the benefit is more pronounced in patients with medium- and low-dose hormone therapy, early administration of hormones, and hormone therapy for more than 7 days. However, no improvement in PaO_2_/FiO_2_ by glucocorticoid treatment was found, which needs to be confirmed by further studies.

## Figures and Tables

**Figure 1:** Flow chart of literature screening.

**Figure 2:** Risk of bias for included studies.

**Figure 3:** Effect of glucocorticoids on mortality of adult ARDS patients.

**Figure 4:** Effects of glucocorticoids on PaO_2_/FiO_2_ in adult ARDS patients.

**Table 1:** Clinical characteristics of the included studies.

Author	Year	Study design	Sample size (hormone group/control group)	The age of the hormone group, years	The age of the control group, years	Hormone group dosing regimen	Treatment time, days
Annane et al. [11]	2006	RCT	85/95	62.0 ± 15.0	58.0 ± 18.0	Hydrocortisone, 50 mg/6h	25
Azevedo et al. [12]	2011	RCT	133/133	57.6 ± 5.2	56.2 ± 4.9	Methylprednisolone, 1 g/d	3
Bernard et al. [13]	1987	RCT	50/49	55.0 ± 2.0	56.0 ± 2.0	Methylprednisolone, 120 mg/d	1
Confalonierid et al. [14]	2005	RCT	23/23	66.6 ± 14.7	60.4 ± 17.3	Hydrocortisone, 240 mg/d	7
Meduri et al. [16]	1998	RCT	16/8	47.0 ± 3.9	51.0 ± 6.6	Methylprednisolone, 2 mg/kg/d	32
Meduri et al. [15]	2007	RCT	63/28	50.1 ± 15.3	53.2 ± 15.3	Methylprednisolone, 1 mg/kg/d	28
Steinberg et al. [17]	2006	RCT	89/91	49.0 ± 19.0	49.2 ± 16.5	Methylprednisolone, 2 mg/kg/d	25
Tongyoo et al. [18]	2016	RCT	98/99	64.5 ± 17.3	64.3 ± 16.0	Hydrocortisone, 50 mg/6h	7
Villar et al. [19]	2020	RCT	139/138	56.0 ± 14.0	58.0 ± 15.0	Dexamethasone, 20 mg/d	10
Wan et al. [20]	2011	RCT	38/43	51.0 ± 15.0	49.0 ± 13.0	Dexamethasone, 1 mg/kg/d	3

RETRACTED

**Table 2:** Subgroup analysis of glucocorticoids on mortality in adult ARDS patients.

Group	Sample size (hormone group/control group)	Events (hormone group/control group)	RR	95% CI	*P*	*I* ^2^ (%)
*Hormone doses*						
Medium and small dose	551/525	152/203	0.73	0.58–0.92	0.007	34
High doses	183/182	50/71	0.70	0.36–1.38	0.31	82

*The start time of hormone therapy*						
Early delivery	468/481	133/193	0.74	0.56–0.99	0.04	55
Late delivery	266/226	69/81	0.68	0.47–0.99	0.05	38

*Duration of hormone therapy*						
Within 7 days	319/324	89/114	0.81	0.57–1.15	0.24	55
More than 7 days	415/383	113/160	0.66	0.50–0.88	0.005	40

## Data Availability

The data used to support the findings of this study are available from the corresponding author upon request.
